RETRACTED

# Akt Inhibition Enhanced the Growth Inhibition Effects of Low-Dose Heavy-Ion Radiation *via* the PI3K/Akt/p53 Signaling Pathway in C6 Glioblastoma Cells

**DOI:** 10.3389/fonc.2021.649176

**Published:** 2021-04-01

**Authors:** Ke Huang, Wei Zhao, Xuqiao Wang, Yingfei Qiu, Zelin Liu, Rui Chen, Wei Liu, Bin Liu

**Affiliations:** ^1^ School/Hospital of Stomatology, Lanzhou University, Lanzhou, China; ^2^ Peking University People’s Hospital, Peking University, Beijing, China; ^3^ Lanzhou University Second Hospital, Lanzhou University, Lanzhou, China; ^4^ The School of Nuclear Science and Technology, Lanzhou University, Lanzhou, China

**Keywords:** heavy-ion radiation, glioblastoma, growth inhibition, perifosine, PI3K/Akt/p53 pathway

## Abstract

**Background:**

Glioma has one of the highest mortality rates of all tumors of the nervous system and commonly used treatments almost always fail to achieve tumor control. Low-dose carbon-ion radiation can effectively target cancer and tumor cells, but the mechanisms of growth inhibition induced by heavy-ion radiation *via* the PI3K/Akt signaling pathway are unknown, and inhibition by heavy-ion radiation is minor in C6 cells.

**Methods:**

Carbon-ion radiation was used to investigate the effects of heavy-ion radiation on C6 cells, and suppression of Akt was performed using perifosine. MTT assays were used to investigate optimal perifosine treatment concentrations. Clone formation assays were used to investigate the growth inhibition effects of carbon-ion radiation and the effects of radiation with Akt inhibition. Lactate dehydrogenase release, superoxide dismutase activity, and malondialdehyde content were assessed to investigate oxidative stress levels. Expression levels of proteins in the PI3K/Akt/p53 signaling pathway were assessed *via* western blotting.

**Results:**

The 10% maximum inhibitory concentration of perifosine was 19.95 μM. In clone formation assays there was no significant inhibition of cell growth after treatment with heavy-ion irradiation, whereas perifosine enhanced inhibition. Heavy-ion radiation induced lactate dehydrogenase release, increased the level of malondialdehyde, and reduced superoxide dismutase activity. Akt inhibition promoted these processes. Heavy-ion radiation treatment downregulated Akt expression, and upregulated B-cell lymphoma-2 (Bcl-2) expression. p53 and Bcl-2 expression were significantly upregulated, and Bcl-2-associated X protein (Bax) expression was downregulated. The expression profiles of pAkt, Bcl-2, and Bax were reversed by perifosine treatment. Caspase 3 expression was upregulated in all radiation groups.

**Conclusions:**

The growth inhibition effects of low-dose heavy-ion irradiation were not substantial in C6 cells, and Akt inhibition induced by perifosine enhanced the growth inhibition effects *via* proliferation inhibition, apoptosis, and oxidative stress. Akt inhibition enhanced the effects of heavy-ion radiation, and the PI3K/Akt/p53 signaling pathway may be a critical component involved in the process.

RETRACTED

## Introduction

Glioma is a neurogliocytic tumor that originates in the brain or spine, and it is one of the most common and deadly tumors of the nervous system (1–4). Current standard treatments for glioma include surgical resection and adjuvant chemotherapy combined with radiation therapy (5). Because of glioma’s high tendency to invade surrounding tissues however, commonly used treatment protocols seldom result in tumor control (6). Due to resistance to chemotherapy and radiation, the malignant nature of glioma results in a high recurrence rate (6). As a direct result, patients with malignant glioma benefit little from standard treatments (7, 8).

Radiation therapy is a relatively standard cancer treatment, and it is generally used to diminish the volume of the neoplasm and increase the effective killing of cancer cells. Substantial therapeutic effects of carbon-ion radiotherapy have been demonstrated in a number of high-risk cancers, including malignant salivary gland tumors, malignant melanoma, and adenocarcinomas of the head and neck region (9, 10). Carbon-ion radiation has numerous effects on cells by breaking chemical bonds in all basic cellular components such as DNA, and ^12^C^6+^ ions generate high relative biological efficiency and steep lateral dose gradients between the target tissues and surrounding areas by reducing lateral scattering (11–14). In a previous study that evaluated the tumor microenvironment and x-ray or carbon-ion radiation of C6 cells, carbon-ion radiation was superior to x-rays for inhibiting tumorigenesis (15). Despite the fact that heavy-ion radiotherapy has a greater capacity to target cancer and is associated with less injury to the surrounding normal tissues, the mechanisms involved in the growth inhibition effects are unknown.

Abnormal activation of the PI3K/Akt pathway is related to cell proliferation and survival in different cancers and tumors (16, 17), and Akt overexpression is associated with resistance to chemotherapeutic agents (18). There are few reports on relationships between the PI3K/Akt signal pathway and the growth inhibition effects of radiation however, and whether the novel Akt inhibitor perifosine can enhance this inhibition warrants further investigation (19). In the present study the effects of heavy-ion radiation on the cell growth, oxidative stress, and relevant signal pathways in C6 cells were investigated, as were the effects of perifosine on the inhibition of growth by heavy-ion radiation.

RETRACTED

## Materials and Methods

### Cell Culture

C6 glioblastoma cells were obtained from the Cell Bank of the Chinese Academy of Sciences (Shanghai, China) and cultured in Dulbecco’s Modified Eagle’s Medium (Gibco, USA) supplemented with 10% (v/v) fetal bovine serum (ABW, Shanghai, China), 100 U/ml penicillin, and 100 μg/ml streptomycin (Basal Media, Shanghai, China). The cells were maintained in logarithmic phase by seeding at a concentration of 5 × 10^4^/ml. After cell confluence reached 70–80% the cells were subcultured at the same concentration. When consistent cell growth was evident, experiments were conducted.

### Heavy-Ion Irradiation

Carbon-ion irradiation was performed at the Heavy-ion Research Facility in Lanzhou (Institute of Modern Physics, Chinese Academy of Sciences, Lanzhou, China). C6 glioblastoma cells were exposed at a dose rate of 0.5 Gy/min using an 80.55-MeV/u ^12^C^6+^ beam. The calculated dose was based on the following previously described formulation (20), in which D is the irradiation dose, P is the ion flux (ions/cm^2^), *ρ* is the medium absorption index (*ρ*_water_ = 1), and dE/dx is the energy loss given by a charged particle in water (keV/µm):

$$\text{D}(\text{Gy})=1.602\times 10^{-9}\times \text{P}\times \left(\text{dE}/\text{dx}\right)\times \rho^{-1}$$

The cells were incubated in fresh complete media for 24 h prior to irradiation, with or without 19.95 μM perifosine. The heavy-ion radiation doses assessed were 0.0, 0.5, 1.0, and 2.0 Gy.

### MTT Assay

MTT assays (21) were used to evaluate cell viability and the cytotoxicity of perifosine (AbMole, USA), so as to determine the optimal treatment concentration of perifosine. C6 cells were seeded in a 96-well plate at a density of 5,000 cells/well and incubated overnight in a humidified incubator (37°C, 5% CO_2_). Adherent cells were then exposed to various concentrations of perifosine for 24 h. The highest concentration of perifosine assessed was 1,600 μM, and successive two-fold dilutions thereof were also assessed (**Figure 1**). After drug exposure, 20 μl MTT working solution was added into each well (MTT final concentration 0.5 mg/ml). After incubation for 4 h, the supernatant was replaced with 150 μl dimethylsulfoxide (Solarbio, Beijing, China), and the plate was incubated in a constant temperature shaker (150 r/min, 37°C) for 15 min. Absorbance was measured at 570 nm using a microplate reader (Infinite^®^ M200 Pro, Tecan Group, Switzerland). Cell survival was calculated *via* the following formula:

$$\text{Survival rate}=\left({\text{OD}}_{\text{treatment group}}/{\text{OD}}_{\text{control group}}\right)\times 100\%$$

**Figure 1:** Growth inhibition perifosine dose–response curve in C6 cells. The MTT assay was used to measure cell viability, and the 10% maximum inhibitory concentration of perifosine was 19.95 μM. Survival rate = (OD_treatment group_/OD_control group_) × 100%.

RETRACTED

### Clone Formation Assay

Clone formation assays were performed to determine the effects of carbon-ion irradiation and the effects of perifosine. Cell suspensions were plated in 60-mm culture dishes pretreated with 0.1% polylysine (Solarbio) at a density of 1,000 cells per dish. The dishes were then exposed to the doses of carbon-ion radiation described in the *Materials and Methods* section. After incubation at 37°C for 12 days in a humidified incubator containing 10% CO_2_ the plates were stained with 0.1% Giemsa (Sigma, Shanghai, China) for 10 min. After washing with slow-running ultra-pure water for 5 min, the results were processed using ImageJ software (v. 1.47, Wayne Rasband, National Institutes of Health, USA). The number of cell clones containing more than 50 cells was counted. The colony formation rate of each group was calculated as the number of cell clones divided by the number of inoculated cells, expressed as a percentage.

### Lactate Dehydrogenase, Superoxide Dismutase, and Malondialdehyde

Lactate dehydrogenase (LDH) release, superoxide dismutase (SOD) activity, and malondialdehyde content were assessed *via* colorimetric assays, as measures of oxidative stress. Three days after irradiation the supernatant of the culture medium was collected, and LDH release was measured using a commercially available LDH assay kit (Nanjing Jiancheng, Nanjing, China) in accordance with the manufacturer’s instructions. SOD activity and malondialdehyde content in cells were assessed *via* SOD assay kits and malondialdehyde assay kits (Nanjing Jiancheng).

### Hoechst 33258 Staining

In order to investigate the cells’ apoptosis, morphological analysis was performed by Hoechst 33258 staining. C6 cells were seeded in 24-well culture plate at a density of 5 × 10^4^ cells per well. The cells were then exposed to the doses of carbon-ion radiation described in *Heavy-Ion Irradiation* section. After incubation at 37°C for 24 h in a humidified incubator containing 10% CO_2_, the cells were stained with Hoechst 33258 (Solarbio) for 20 min, followed by observation under a fluorescence microscope. Strong fluorescence can be observed in the nuclei of apoptotic cells, while weak fluorescence was observed in non-apoptotic cells.

### Caspase-3 Activity

Caspase-3 activity was estimated using Caspase-3 assay kit (Abcam, UK). Absorbance was measured at 405 nm using a microplate reader (Infinite^®^ M200 Pro).

RETRACTED

### Western Blotting

Relative expression of proteins involved in PI3K/Akt/p53 signaling pathways was assessed *via* western blotting. After irradiation with or without perifosine and a subsequent 72-h incubation, RIPA Lysis Buffer (Solarbio) containing 1.0% phenylmethylsulfonyl fluoride (Solarbio) was used to extract total protein from the samples. Protein concentrations were then measured *via* the BCA Protein Assay Kit (CWBIO, Beijing, China). Equal amounts of protein were loaded onto SDS−PAGE gels (Solarbio) for protein separation, then the proteins were transferred onto polyvinylidene fluoride membranes (Millipore, USA). After blocking with 5% non-fat milk (BD, USA) for 1 h at room temperature the membranes were incubated overnight at 4°C with primary antibodies in a constant temperature shaker (60 r/min, 4°C). The primary antibodies used were Ras (Abcam) at 1:1,000, total Akt (CST, USA) at 1:800, pAkt (CST) at 1:800, p53 (CST) at 1:800, B-cell lymphoma-2 (Bcl-2) (Abcam) at 1:1,000, Bcl-2-associated X protein (Bax) (Abcam) at 1:1,000, caspase 3 (Abcam) at 1:1,000, and glyceraldehyde 3-phosphate dehydrogenase (Abcam) at 1:1,000. After washing the membranes in Tris-buffered saline containing 0.05% Tween 20, they were then incubated with the secondary antibody (Proteintech, Wuhan, China) for 2 h. Lastly, after washing the membranes, ECL chemiluminescence reagents (Amersham Pharmacia Biotech, Japan) were used to visualize the proteins. Quantity One software (v. 4.6.2, Bio-Rad, Hercules, CA, USA) was used to quantify band intensities. Relative protein expression was normalized to glyceraldehyde 3-phosphate dehydrogenase.

### Statistical Analysis

Data were assessed *via* one-way analysis of variance using GraphPad Prism software (v. 8.3.0, La Jolla, CA, USA) and SPSS (v. 21.0, Chicago, IL, USA), and are represented as means ± the standard deviation. *p* <0.05 was deemed to indicate statistical significance.

## Results

### Growth Inhibition Induced by Heavy-Ion Radiation, and Effects of Akt Inhibition

Cell growth inhibition was measured *via* the MTT assay, to determine the optimal treatment concentration of perifosine. A concentration–response curve was generated using GraphPad Prism software, and the 10% maximum inhibitory concentration of 19.95 μM was identified using SPSS (**Figure 1**). In a subsequent clone formation assay, at a perifosine concentration of 19.95 μM, there was no significant difference between the perifosine group and the control group (*p* > 0.05) (**Figure 2**). Based on the above results, a perifosine concentration of 19.95 μM was used in subsequent experiments.

RETRACTED

**Figure 2:** **(A)** Representative images showing colonies formed in different groups. **(B)** Quantitative analysis of the numbers of colonies formed by different groups of cells. Data shown are means from three independent experiments. *p < 0.05 *vs.* control or other groups.

The effects of carbon-ion irradiation on C6 cells with and without Akt inhibition were investigated using a plate clone formation assay, and there was no significant inhibition of cell growth after treatment with heavy-ion irradiation. Conversely, perifosine treatment significantly enhanced the growth inhibition effects of irradiation at doses of 1.0 and 2.0 Gy (*p* < 0.05) (**Figure 2**). In contrast to a previous study (22), the same irradiation treatments were applied to Hela cells without perifosine, and the growth inhibition was more pronounced (**Figure 3**).

**Figure 3:** Quantitative analysis of the numbers of colonies formed by different groups of cells. Data shown are means from three independent experiments. Hela data are from Liu et al. (21). *p < 0.05 *vs.* control or other groups.

### Oxidative Stress Imbalance Induced by Heavy-Ion Irradiation, and Effects of Akt Inhibition

To determine whether ^12^C^6+^ ionizing radiation induced the imbalance in oxidative stress and whether perifosine facilitated this process, LDH, SOD, and malondialdehyde levels were measured. LDH release and malondialdehyde content were upregulated after carbon-ion irradiation, whereas SOD activity was downregulated (**Figure 4**). There were no significant differences between groups irradiated without perifosine (*p* > 0.05). In contrast, perifosine treatment significantly increased LDH and malondialdehyde levels, and reduced the level of SOD when the radiation dose was increased to 1.0 or 2.0 Gy (*p* < 0.05).

**Figure 4:** **(A, B)** An oxidative stress imbalance was induced by heavy-ion radiation, and the imbalance was enhanced by perifosine. The effects of heavy-ion radiation with and without perifosine on malondialdehyde and SOD in C6 cells were determined using commercial kits. **(C)** An oxidative stress imbalance was induced by heavy-ion radiation, and the imbalance was enhanced by perifosine. The effects of heavy-ion radiation with and without perifosine on LDH release in C6 cells were determined using commercial kits. *p < 0.05 *vs.* control or other groups.

### Effects of Heavy-Ion Irradiation on Apoptosis Pathways

Hoechst 33258 staining is used to visualize condensed nuclei in apoptotic cells and heavy-ion irradiation plus perifosine induced accumulation of apoptotic bodies, whereas the apoptotic response was low when cells were treated with heavy-ion irradiation without perifosine (**Figure 5**). Caspase-3 activity was robustly upregulated after heavy-ion irradiation plus perifosine treatment (**Figure 6**), which is corresponding to the former results. The western blotting analysis shows that Bcl-2 expression was significantly upregulated by heavy-ion irradiation, and Bax expression was downregulated. These effects were reversed when the cells were treated with perifosine. Increases in caspase 3 expression were observed in all radiation groups, and these increases were more pronounced when the cells were treated with perifosine (**Figure 7**).

RETRACTED

**Figure 5:** After heavy-ion irradiation with or without perifosine, cells were stained with Hoechst 33258, and abundant apoptotic bodies were observed in perifosine treated groups.

**Figure 6:** After heavy-ion irradiation with or without perifosine, Caspase-3 activity in C6 cells was determined using a commercial Caspase-3 assay kit. *p < 0.05 *vs.* control or other groups.

**Figure 7:** After heavy-ion irradiation with or without perifosine, the expression levels of proteins were determined *via* western blotting. Glyceraldehyde 3-phosphate dehydrogenase was used as a loading control. Experiments were repeated three times. Representative images of western blots are shown. *p < 0.05 *vs.* control or other groups.

### Effects of Heavy-Ion Irradiation on PI3K/Akt Pathways

Protein expression levels of Akt were significantly reduced after exposure to different doses of heavy-ion irradiation alone (*p* < 0.05), whereas pAkt and p53 expression were significantly upregulated. Ras expression increased when the cells were irradiated at a dose of 0.5 Gy, but declined at greater heavy-ion irradiation doses. pAkt expression was downregulated after treatment with perifosine (**Figure 7**).

## Discussion

Glioma has one of the highest mortality rates of all tumors of the nervous system, and commonly used treatment protocols seldom lead to tumor control. Carbon-ion radiation generates high relative biological efficiency, and dominant therapeutic effects have been observed. In the current study there was no significant difference after treatment with heavy-ion radiation (**Figure 2**), and a low concentration of perifosine significantly enhanced the growth inhibition effects of radiation at doses of 1.0 and 2.0 Gy, suggesting that Akt inhibition may have the potential to enhance the efficacy of heavy-ion radiotherapy.

Necrotic death can limit cellular growth (23). LDH analysis measures the release of LDH from cells by damaging cell membranes (24), hence in the present study LDH leakage was measured as an indicator of cell necrosis. LDH release levels were consistent with the results of the clone formation assays (**Figures 2**, **4C**). ^12^C^6+^ ionizing radiation induced an increase in LDH release, and perifosine promoted this process. These results suggest that Akt inhibition promotes necrotic death in C6 cells exposed to heavy-ion radiation.

RETRACTED

Oxidative stress plays a key role in the pathogenesis of radiation-induced damage, and cells can rapidly scavenge free radicals and reactive oxygen *via* antioxidants and enzymes under normal physiological conditions to maintain redox system homeostasis (25). Abundant reactive oxygen is constantly produced and accumulated in radiation-induced cell injury. Oxidative stress is induced, and the intracellular oxidant/antioxidant balance is disrupted. Consequently, structural damage to cells and changes in enzyme activity can occur *via* chain reactions (26–28). In the present study, malondialdehyde was upregulated and SOD expression was downregulated, and perifosine treatment significantly strengthened these trends (**Figures 4A, B** **)**. These results indicate that disordered oxidative stress may account for the killing effect of heavy-ion radiation, and Akt inhibition promotes a vicious cycle of oxidative stress.

Radiation-induced apoptosis has been reported (29). In the mitochondrial pathway, Bcl-2 is a major protein that inhibits apoptosis, whereas the central cell death regulator Bax induces apoptosis (26). These proteins also regulate cell death signaling pathways and are involved when various signals converge (30). The apoptosis-related protein caspase 3 is essential for morphological changes and DNA fragmentation associated with apoptosis (31, 32). The Hoechst 33258 staining and the measurement of Caspase 3 activity confirmed the apoptotic effects of heavy-ion radiation. The western blotting analysis in the current study indicated that carbon-ion radiation upregulated Bcl-2 expression and downregulated Bax expression, and these effects were reversed by perifosine. An upward trend in caspase 3 expression was observed in all radiation groups, and the trend was more pronounced in perifosine-treated groups. These results indicate that Akt inhibition may enhance the killing effects of heavy-ion radiation.

The PI3K/Akt/p53 signaling pathway is known to be active in numerous tumors, and is involved in cell death, survival, and apoptosis (19, 33–35). RAS may function upstream of PI3K/Akt signaling pathways to regulate tumor development (36). Activation of p53, a protein downstream of the PI3K/Akt signaling pathway, may lead to reversible cell-cycle arrest and protect cells against DNA damage and apoptosis (37, 38). In the current study, heavy-ion radiation upregulated the PI3K/Akt signaling pathway. Moreover, the upstream signal RAS and the downstream signal p53 were upregulated in radiation groups, which may account for the growth inhibition effects of heavy-ion radiation. In contrast, perifosine enhanced the inhibitory effects of heavy-ion radiation.

RETRACTED

## Conclusion

In the present study the growth inhibition effects of heavy-ion radiation were not pronounced in C6 cells, and Akt inhibition enhanced inhibitory effects *via* induction of necrotic cell death, apoptosis, and oxidative stress. Mitochondrial pathways and apoptosis pathways may be involved in heavy-ion resistance. Further research should be undertaken to investigate the role that Akt inhibition plays in heavy-ion radiation treatment.

## Data Availability Statement

The original contributions presented in the study are included in the article/supplementary material. Further inquiries can be directed to the corresponding authors.

## Author Contributions

KH, WL, and BL: conception and design. KH, BL, and ZW: administrative support. KH, WZ, XW, YQ, ZL, and RC: experimental testing. KH, WZ, XW, YQ, ZL, and RC: data analysis and interpretation. All authors contributed to the article and approved the submitted version.

## Funding

This project was supported by the Open Subject Foundation of Key Lab of Oral Diseases of Gansu Province, Northwest Minzu University (Grant No. SZD201901), the Fundamental Research Funds for the Central Universities (Grant No. 31920170196), and Gansu Health and Research Plan Project Funds (Grant No. GSWSKY2017-46), the Postdoctoral Science Foundation of China (Grant No. 22019M653474) and the Projects of Heavy Ion Research Facility in Lanzhou (Grant No. HIR20PY012).

## Conflict of Interest

The authors declare that the research was conducted in the absence of any commercial or financial relationships that could be construed as a potential conflict of interest.
